The article "Literature Review on the Applications of Machine Learning and Blockchain Technology in Smart Healthcare Industry: A Bibliometric Analysis" was retracted in 2023. Reasons: unreliable results or conclusions; concerns about the data; concerns about the peer review; concerns about the citations.

# Literature Review on the Applications of Machine Learning and Blockchain Technology in Smart Healthcare Industry: A Bibliometric Analysis

**DOI:** 10.1155/2021/9739219

**Published:** 2021-08-13

**Authors:** Yang Li, Biaoan Shan, Beiwei Li, Xiaoju Liu, Yi Pu

**Affiliations:** School of Management, Jilin University, Changchun 130022, China

## Abstract

The emergence of machine learning (ML) and blockchain (BC) technology has greatly enriched the functions and services of healthcare, giving birth to the new field of “smart healthcare.” This study aims to review the application of ML and BC technology in the smart medical industry by Web of Science (WOS) using bibliometric visualization. Through our research, we identify the countries with the greatest output, the major research subjects, funding funds, and the research hotspots in this field. We also find out the key themes and future research areas in application of ML and BC technology in healthcare area. We reveal the different aspects of research under the two technologies and how they relate to each other around five themes.

## 1. Introduction

With the revolution of the medical infrastructure in the recent years, the smart healthcare system has been paid more considerable attention [1]. Smart healthcare is a novel concept that refers to a set of rules that integrate prevention, diagnosis, treatment, and management. Different from traditional medical systems, smart medical systems can connect and exchange information at any time and place [2].

Compared with traditional medical treatment, smart healthcare has the characteristics of preventability, immediacy, and interconnection of information. Through wireless network, using portable mobile devices, medical staff can constantly perceive, process, and analyze major medical events (preventability). Doctors can grasp the case information of each patient at any time and quickly develop a diagnosis and treatment plan (immediacy). Medical personnel can log in the medical system anywhere to inquire about medical images and medical advice and patient's referral information can be accessed at any hospital through the medical network (interconnection of information). These functions are supported by new digital technologies. BC follows absolute privacy rules to identify users related to transactions. It is mainly used for the management of information systems to help achieve secure storage, transactions, process automation, and other applications [3]. ML is the leading technology for performing complex analysis, intelligent judgment, and creative problem solving in healthcare [4].

Generally, previous studies related to application of digital technologies in smart healthcare domain were limited to study in one field or one country. No studies have mapped the current status of these two technologies in the medical field. Also, there is no relative study that specifically addresses the relationship between authors, affiliations, keywords, and the hotpots of the research. In the past five years, the study of smart healthcare has attracted extensive attention from scholars of a series of disciplines, which requires us to integrate the viewpoints of scholars of different disciplines and study the status to seek deeper discoveries.

The article "Literature Review on the Applications of Machine Learning and Blockchain Technology in Smart Healthcare Industry: A Bibliometric Analysis" was retracted in 2023. Reasons: unreliable results or conclusions; concerns about the data; concerns about the peer review; concerns about the citations.

Therefore, this research proposed portraying the status of application of two types of digital technologies, ML and BC, in smart healthcare studies by bibliometric visualization. In this paper, we have presented a comprehensive review on the application of ML and BL techniques in the healthcare sector. We analyze the research status in terms of countries, institutions, publication volume, authors, journals, sponsors, and subject areas. In addition, this paper subdivides the main application scenarios of the prior art in the medical field. Our research will provide healthcare practitioners with an insight to keep ML and BC technologies fully utilized. Finally, we analyze the latest research trends based on ML and BC technology in order to provide a research direction for future research.

## 2. Methodology

### 2.1. Research Method

This study mainly applied bibliometrics to conduct a comprehensive analysis of the articles published on WOS related to the application of machine learning and blockchain technology in the field of smart healthcare. Bibliometric analysis makes a visual analysis of the research field by analyzing the information obtained from the database, such as titles, abstracts, keywords, and references. Bibliometric analysis helps researchers review a research area more scientifically and systematically and discover future research trends [5]. Since WOS contains scientific literature of all disciplines, our literature collection process is carried out in Web of Science [6].

### 2.2. Research Process

Our research process is divided into four steps: problem formulation, literature search, basic analysis, and VOSviewer analysis.

1. Problem formulation: Our study aims to provide a comprehensive presentation of the application of ML and BC in the field of smart medicine by visualizing existing publications. To achieve this goal, we developed and solved the following research questions: How much attention have scholars paid to emerging technologies and smart medicine in recent years? What are the representative literatures? What are the current research topics and how are they evolving?
2. Literature search: Literature search is divided into two steps: subject word search and manual screening. The first step is subject word search in the Web of Science core data set using the retrieval formula TS = (“machine learning” OR “blockchain”) AND TS = (“smart healthcare”). The first round of screening finally obtained 118 documents (data gathering took place in May 2021). The second step is manual literature screening. Our purpose is to eliminate the document that is not relevant to this field and to obtain the research direction and research progress in this field more accurately. The team members carefully read the titles, keywords, and abstracts of 118 documents and scanned the full text when necessary to ensure the relevance of the document. Finally, 112 documents were obtained as our research objects.
3. Basic analysis: Basic analysis refers to the analysis results that can be directly exported from the WOS database or can be obtained through statistics. We conducted a statistical analysis of the year in which the literature was published, the research field, the fund sponsor, and so on. Through basic analysis, researchers can gauge changes in scholars' and institutions' interest in research in the field and understand research trends.
4. VOSviewer analysis: VOSviewer analysis is to use VOSviewer to build a bibliometric network. We listed the most influential authors and literature in the field and showed heat maps of keyword research. We also used a clustering technique based on keywords cooccurrence to study the conceptual structure and distinctive clusters of a research field [7].

The article "Literature Review on the Applications of Machine Learning and Blockchain Technology in Smart Healthcare Industry: A Bibliometric Analysis" was retracted in 2023. Reasons: unreliable results or conclusions; concerns about the data; concerns about the peer review; concerns about the citations.

## 3. Result

### 3.1. Number of Documents per Year

Research on this topic first appeared in the WOS database in 2015 (Figure 1). In 2015, Tucker et al. [8] published an article titled “*Machine learning classification of medication adherence in patients with movement disorders using non-wearable sensors*” in *Computers in Biology and Medicine*. This paper demonstrates that nonwearable hardware and data mining models can be used to monitor medication compliance outside of traditional healthcare settings. It has initiated the research of machine learning in the field of intelligent medicine and laid a foundation for later research.

The number of international documents on smart healthcare study is increasing year by year (Figure 1). The peak number of articles was 54 in 2020, double the number of articles published in 2019. This study finds that there are three reasons for the rapid growth of publications. First, the demand for applications in the medical industry has been growing with the data-intensive development of smart applications, and the market for smart medicine is gradually expanding [9]. Second, more and more international researchers (such as Venkatesan et al. [10]) began to study the application of blockchain and machine learning in the field of intelligent medicine. Finally, more and more journals such as *Sensors* are more willing to accept research related to this field.

The article "Literature Review on the Applications of Machine Learning and Blockchain Technology in Smart Healthcare Industry: A Bibliometric Analysis" was retracted in 2023. Reasons: unreliable results or conclusions; concerns about the data; concerns about the peer review; concerns about the citations.

### 3.2. Major Research Subject Areas

Figure 2 shows the subject area with the widest application of machine learning and blockchain in smart healthcare research is Computer Science, with 76 documents (33.33%). The second major research area is Engineering with 66 documents (28.95%), and Telecommunications ranked third with 47 documents (20.61%). An article may cover multiple subject classifications. As for the application of machine learning and blockchain technologies in the field of intelligent medicine, the vast majority of researches start from the technical perspective, such as Computer Science, Engineering, and Telecommunications. However, there were only three articles related to biochemistry, such as Health Care Sciences & Services, accounting for 1% of the total literature. This indicates that the application of blockchain technology and machine learning technology in the healthcare field is still in the experimental stage of technology research and development, and the application of technology is not mature and widespread.

### 3.3. Sponsoring Funding

Figure 3 shows the main funders to help publish research on the application of ML and BC technologies in smart healthcare are the National Natural Science Foundation with 8 papers, the European Commission with 6 papers, and King Saud University with 5 papers. This result is directly related to the number of articles published in China. According to the funding of various institutions, China attaches great importance to the application of machine learning and blockchain in the field of smart health.

### 3.4. Countries

The countries with the highest number of publications of smart healthcare research are India and China, with 23 documents each (Figure 4). It was followed by Saudi Arabia with 22 documents, South Korea with 17 documents, the United States with 15 documents, and Pakistan with 12 documents (Figure 4 shows the number of documents issued by all the issuing countries). It is reasonable considering the population size of India and China. Asian countries publish more articles than European regions.

India, China, Saudi Arabia, and other countries have published more documents in the field of smart medicine, which can be explained from three aspects. First of all, the medical level of developing countries such as India, China, and Saudi Arabia needs to be improved and they need to rely on new technologies to further improve the efficiency and quality of medical treatment. Secondly, machine learning, blockchain, and other new technologies have wide application markets in China, India, and Saudi Arabia. There is a great demand for new technologies in the medical industry, which provides conditions for technology commercialization. Finally, the large number of documents in countries such as China and Saudi Arabia is also influenced by the funding they received.

The article "Literature Review on the Applications of Machine Learning and Blockchain Technology in Smart Healthcare Industry: A Bibliometric Analysis" was retracted in 2023. Reasons: unreliable results or conclusions; concerns about the data; concerns about the peer review; concerns about the citations.

### 3.5. The Most Cited Papers

The publication of smart healthcare studies with the most 10 citations is listed in Table 1. Referring to the largest number of articles in the first ten articles that appeared in 2005, Tucker et al. have developed a noninvasive sensor to monitor adherence of Parkinson's patients to drugs, by reading data of patients, to distinguish between patients taking their medicine diagnosis and treatment at home and it can realize the early warning and effectiveness of clinical trials as high as 97%.

Through the analysis of the most cited literatures, it is found that the main application of machine learning in the medical field is the diagnosis of diseases in these highly cited articles such as remote healthcare, disease diagnosis, healthcare monitoring, medication adherence, and body sensor. The main application of blockchain in the medical field is data encryption. The article related to blockchain focuses on its role in Multilevel Privacy-Preserving, monitoring patient vital sign, privacy health data, and Drug Supply Chain Integrity Management.

### 3.6. Research Hotspots

Figure 5 is the keyword heat map made according to the keywords in 112 articles. The darker the color, the higher the frequency of the keyword. Through the analysis of the heat map (Figure 5), we found that, in addition to machine learning, blockchain, and smart healthcare, Internet and the Internet of Things are also core keywords of this area.

IoT appears in the keywords because the outbreak of chronic diseases such as Novel Coronavirus has once again aroused the attention to intelligent medical treatment. IoT technology is used to monitor patient's vital sign. Smart healthcare can reply to such complex and urgent medical emergencies and make up for the shortcomings of the original medical system. The Internet of Things enables wearable devices to collect large amounts of data. It is considered as the communication between objects due to being embedded in sensors [11, 12]. The Internet of Things in healthcare connects millions of sensors to a patient's body to continuously monitor his or her physical condition.

## 4. Theme Clustering Analysis

Through the author keywords and keywords plus, we used VOSviewer to construct the keyword network diagram. VOSviewer is a software tool for building and visualizing bibliometric networks that generate clusters that represent the underlying structure of a document. Specifically, we used bibliometric tools to analyze the keywords in articles, extract the most commonly used terms, and map them according to their interrelationships. From this analysis, we can determine the topics that are most commonly used in this field. In 112 articles, a keyword that appears at least three times is required to appear in the keyword network. Therefore, from 582 keywords, there were only 55 keywords that meet the thresholds.  Figure 6 shows that there were five groups of study themes based on research keywords related to the study. Large circles indicate terms that are used more frequently, and color-coded lines indicate cooccurrence of terms. We found that the circles of the same color might come from a single document, so we read the full text of the documents mapping circles of the same color to see how they fit together. We name the clustering results according to the technical similarity.

The article "Literature Review on the Applications of Machine Learning and Blockchain Technology in Smart Healthcare Industry: A Bibliometric Analysis" was retracted in 2023. Reasons: unreliable results or conclusions; concerns about the data; concerns about the peer review; concerns about the citations.

### 4.1. Cluster 1: Machine Learning

Cluster 1 is what we call Machine Learning (red). The keywords for this topic were smart healthcare, machine learning, biomedical monitoring, data analytics, data mining, deep learning, fusion, human activity recognition, model, medical diagnostic imaging, neural network, and smart home.

Machine learning, a field of artificial intelligence, has been widely used in the medical industry. With the development of ICT technology and the arrival of the era of big data, information such as patient information, medical treatment records, and medication status has been digitized, and a large amount of data has been generated in the field of medicine and healthcare [13]. The medical industry uses machine learning to deeply analyze complex medical data, which has become the main direction of machine learning research.

Cluster 1 centers around the application of machine learning in the medical field. Specifically, the research focuses on how the medical industry uses machine learning methods such as deep learning, neural network learning, and feature fusion to realize data analysis and mining. The goal is to realize the identification of human activities, health monitoring, disease prediction, and diagnosis and promote the development of the field of smart medicine.

Gumaei et al. [14] applied machine learning to human activity recognition. They proposed a human activity recognition framework based on multisensor hybrid deep learning model. This method can process multisensor data more intelligently and help medical institutions better care for the elderly and patients. Souri et al. [15] applied machine learning to the student health monitoring system, collected data through the Internet of Things, and analyzed data through machine learning to continuously monitor the physical condition of students. Ali et al. [16] built a disease prediction system based on deep learning feature fusion and information gain technique to predict the incidence of heart disease and create conditions for the effective treatment of patients with heart disease. Chui et al. [17] reviewed previous research on disease diagnosis in the field of intelligent medicine, summarized emerging machine learning algorithms, and discussed the challenges of deploying disease diagnosis in the future.

The article "Literature Review on the Applications of Machine Learning and Blockchain Technology in Smart Healthcare Industry: A Bibliometric Analysis" was retracted in 2023. Reasons: unreliable results or conclusions; concerns about the data; concerns about the peer review; concerns about the citations.

### 4.2. Cluster 2: Artificial Intelligence

When exploring the second group, Artificial Intelligence cluster (green), there were items like architecture, cloud computing, edge, edge computing, fog computing, medical services, pathology, and smart city.

Artificial intelligence refers to the intelligence shown by machines made by people. In general, artificial intelligence refers to the technology that represents human intelligence through ordinary computer programs. In the field of computer, artificial intelligence has been paid more and more attention; and, in the robot, economic and political decision-making, control system, and simulation system have been applied. Artificial intelligence is also getting more and more attention in the medical field.

Cluster 2 focuses on the application of artificial intelligence in the field of intelligent medicine. Specifically, the role of artificial intelligence is mainly reflected in the analysis and processing of data generated by intelligent devices such as the Internet of Things and sensors.

Artificial intelligence is attracting more and more attention in the medical field [18, 19], and it is mostly used to assist decision-making in the medical field. Kamruzzaman [18] found that AI systems could be used for ancillary medical care by processing data from patients who admitted to hospital for emergency treatment or providing early detection of major diseases. With the assistance of artificial intelligence, the patient's human body data and genetic data can be automatically analyzed and generated medical reports to provide decision support to doctors. The reason why artificial intelligence can assist decision-making is the huge growth of medical data analysis and research. On the one hand, it can increase the accuracy and timeliness of decision-making, and, on the other hand, it can greatly alleviate the shortage of medical resources (medical staff and equipment) and save costs. Chui et al. [19] applied artificial intelligence to a particular disease for three kinds of detection of speech disorders.

The article "Literature Review on the Applications of Machine Learning and Blockchain Technology in Smart Healthcare Industry: A Bibliometric Analysis" was retracted in 2023. Reasons: unreliable results or conclusions; concerns about the data; concerns about the peer review; concerns about the citations.

### 4.3. Cluster 3: Blockchain

The third group of keywords, Blockchain cluster (yellow), includes access control, cloud, electronic medical records, Ethereum, privacy, security, and smart contracts.

Blockchain technology refers to a distributed, decentralized, and immutable digital ledger that records transactions through a global computer network, in which the information is highly secure [20]. It has grown into a very rich and efficient technology to serve and instruct the healthcare patient's point of view, to maintain patient data privacy, and to provide physicians with real-time, accurate, and trusted data of the process [21].

Cluster 3 revolves around the application of blockchain in the field of smart medicine. Specifically, the role of blockchain in the medical field is divided into two categories, the first category revolves around the encryption of medical data generated by individual patients, and the other category is applied to the supply chain system management of drugs. As the scalability of wearable medical devices increases, the smart medical field faces challenges in maintaining privacy and security. Scholars are building different frameworks for blockchain to improve the security of medical data.

In addition, blockchain technology can also assist in decision-making. Gul et al. [22] proposed an intelligent medical business model based on blockchain, which is customer-centered business. On the other hand, blockchain technology is applied in the drug supply chain management, supply chain involves a certain degree of stakeholders, and one of the biggest challenges associated with the supply chain is temperature monitoring and preventing fake drugs. Singh et al. [23] proposed a blockchain framework based on IoT sensors to track the movement of drugs in the supply chain. The safety of the pharmaceutical supply chain has become a major public health concern, and this is a collective process [24].

### 4.4. Cluster 4: Sensor Cluster

Sensor cluster (purple) was dominated by the keywords sensor, feature extraction, activity recognition, classification, prediction, smart healthcare system, care, and healthcare.

Sensor technology, communication technology, and computer technology together form the three pillars of modern information technology. With the development of sensor technology, sensors are becoming more and more intelligent and widely used. Sensors can collect data in real time. By analyzing the collected data, targets such as tracking patients' physical conditions, taking medicines, and identifying activities can be realized [25]. The application of sensors has greatly improved the quality and efficiency of the medical industry and reduced the cost of treatment, so it is widely used in the medical field.

The article "Literature Review on the Applications of Machine Learning and Blockchain Technology in Smart Healthcare Industry: A Bibliometric Analysis" was retracted in 2023. Reasons: unreliable results or conclusions; concerns about the data; concerns about the peer review; concerns about the citations.

Cluster 4 focuses on the application of sensors in the field of smart healthcare. Specifically, Cluster 4 mainly studies the method of using sensors to collect data in the medical industry, using feature extraction technology to extract data features, and realizing activity recognition and state prediction through classification algorithm. Since data collection in the medical industry mainly relies on sensors and big data is the basis of realizing smart medicine, sensors play a vital role in the process of smart medical industry.

By analyzing data collected from nonwearable multimodal sensors, Tucker et al. [8] modeled and predicted patients' adherence to medication after leaving the clinic. The method can give early warning to the patient's safety status in time and prompt the patient to take the medicine on time. Syed et al. [26] placed multiple wearable sensors on the left ankle, right arm, and chest of the tester, using related technologies to identify the movement of different body parts and determine the type of movement. This method is a good way to remotely monitor the activity status and health status of the elderly. Alo et al. [27] argued that current activity identification methods are not good at analyzing complex and dynamic activities. Therefore, a deep stacked autoencoder algorithm is proposed for the smartphone-embedded accelerometer sensor data, which can automatically extract the data features and improve the accuracy of activity recognition. Khan et al. [28] believed that wearable devices with embedded sensors can record data but have limitations such as battery life and hardware cost. Therefore, the authors further propose that channel state information can be used instead of wearable sensor devices to collect data to predict the health status of patients.

### 4.5. Cluster 5: IoT Cluster

IoT cluster (blue) was related to the keywords authentication, COVID-19, efficient, big data, industries, Internet, and network.

Industry 5.0 is the Fifth Industrial Revolution consisting of intelligent digital information and manufacturing technology [29]. The Fifth Industrial Revolution has promoted the wide application of technologies such as the Internet of Things (IoT). The IoT combines information sensing devices with the Internet, enabling people, machines, and things to get rid of the limitations of time and space and realize interconnection. The rapid development of the IoT has created opportunities for providing personalized services in the medical field [30].

The article "Literature Review on the Applications of Machine Learning and Blockchain Technology in Smart Healthcare Industry: A Bibliometric Analysis" was retracted in 2023. Reasons: unreliable results or conclusions; concerns about the data; concerns about the peer review; concerns about the citations.

Cluster 5 centers on the application of the IoT in the field of smart healthcare. Research topics can be specifically divided into two categories. The first category focuses on how the medical industry applies IoT technology to epidemic prevention and control and patient treatment during the epidemic period. The IoT has the advantage of usability and accessibility, which makes data security a challenge while providing convenience. The second category of research focuses on the security of open data in the IoT and how to protect the data with technologies such as blockchain.

At the beginning of COVID-19, the most effective way to prevent the spread of the virus was to keep a physical distance and wear a mask. In order to effectively monitor the physical distance, Vedaei et al. [31] proposed a system composed of an IoT node, a smartphone application, and machine learning tools. The system records the user's health index, displays his or her health status, and prompts the user about a safe physical distance. In the environment of IoT, data security and information privacy are also concerned. Wazid et al. [32] proposed a blockchain-based secure authentication key management scheme to ensure the security of communication data. Wang et al. [33] invented the GuardHealth system, which can not only realize the sharing of medical data but also guarantee the privacy of medical data. Tahir et al. [3] proposed a blockchain-based network authentication framework for the IoT using a probabilistic model to enhance access control. It can be seen that the security management authentication and access control of the IoT are closely related to blockchain.

The study found that the emergence of these five types of research is based on modern technology and the environment on the existing healthcare services put forward new requirements. The first is the accuracy of data collection, which makes the medical system reliable and effective (sensors), and the second is that patient treatment requires continuous testing and analysis of medical data under different monitoring data, resulting in a large amount of data. How to analyze this data has become a huge challenge (machine learning). The third is the effectiveness of treatment (AI); the need for patient numbers, types of analysis, and response times has become more urgent, new treatments need to be simulated in a robust, and scalable framework that delivers the highest quality results in the shortest possible time. The fourth is the confidentiality of data (blockchain), which is sensitive because it can be maliciously used by terrorists or pharmaceutical monopolists against specific sectors. This requires that such a framework be tamper-proof and nonhackable, preventing any fraudulent manipulation of sensitive medical data. The Internet of Things is the interconnection between medical devices.

The article "Literature Review on the Applications of Machine Learning and Blockchain Technology in Smart Healthcare Industry: A Bibliometric Analysis" was retracted in 2023. Reasons: unreliable results or conclusions; concerns about the data; concerns about the peer review; concerns about the citations.

## 5. Future Research of Machine Learning and Blockchain Technology

After that, we continued to use the authors' keywords to conduct analysis with the help of the software VOSviewer. The lighter the color, the newer the research, and we tried to find and explain this research trend through the color.  Figure 7 shows the trend of the research topic over time; the lighter the color, the newer the research.

### 5.1. Biomedical Monitor

In the research on machine learning, scholars currently monitor and diagnose hormone indicators of chronic diseases (diabetes, Alzheimer's disease, cognitive impairment, etc.) through different algorithms and try to improve the accuracy of monitoring and diagnosis through methodology. Future research will focus on biological monitoring.

Tchito Tchapga et al. [34] have begun to discuss the impact of the size of the data set on machine learning algorithms and have proposed the Spark algorithm to perform the classification of biomedical images. Zhao et al. [35] designed an intelligent disease recognition algorithm based on deep learning algorithm, which has good international adaptability and science for monitoring the adaptive behavior of children with ADHD. Wu et al. [36] have been able to evaluate videos through in-depth learning.

### 5.2. Fog Computing

The Internet of Things (IoT) is facing challenges due to the explosive growth of devices and the amount, variety, accuracy, and speed of the data these devices generate. This requires ultralow latency, reliable service, and security and privacy. Fog computing is a promising solution to overcome these challenges. Fog computing is a highly virtualized technology that provides computing, storage, and networking services in multiple application domains.

The combination of IoT devices and cloud services became the basis of fog computing. Smart medicine promises a health system that connects people and medical institutions in an intelligent way by using technologies such as wearables and IoT devices to access information in real time to deliver healthcare services. A computational distributed fog computing approach processes data from dementia and COPD patients' perceptions in the home environment and sends it to physicians to help them make quick decisions in the comfort of their homes in order to better treat patients with Parkinson's disease [37]. Fog computing is emerging as a key enabler of smart healthcare to ensure adequate patient safety. Fog computing nodes form a distributed network. Blockchain technology is a trusted shared distributed decentralized database archiving technology that caches transaction records across the network and can be easily integrated with fog computing. Tuli et al. proposed another blockchain-based security framework that integrates sensor FOG nodes and cloud servers. Their framework ensures reliability security and QoS [9].

The article "Literature Review on the Applications of Machine Learning and Blockchain Technology in Smart Healthcare Industry: A Bibliometric Analysis" was retracted in 2023. Reasons: unreliable results or conclusions; concerns about the data; concerns about the peer review; concerns about the citations.

### 5.3. Activity Cognition

Sensors can realize the recognition of activities and state prediction through feature extraction, with the assistance of classification algorithm. At present, the application of smart medical systems is still in the initial stage, in which data collection and feature extraction are the key to deploy smart medical infrastructure. Sensors are the foundation of all medical data collection, and one direction for future research is to improve the performance of complex human activity recognition frameworks. The scholars further proposed that channel state information could be used instead of wearable sensor devices to collect data, and feature selection algorithm and classification algorithm could be used to select and classify features, so as to predict the health status of patients.

### 5.4. Security and Privacy

The Internet of Things can provide a new turning point by facilitating communication with nearby entities or objects. Through the Internet of Things, existing research allows doctors and other healthcare personnel to know the status of patients. It can also be stored in a database for further access and can be analyzed so that any serious problems can be prevented or cured if they occur. However, the front-end devices of the Internet of Things, such as temperature sensors, card readers, wearable devices, mobile phones, and other embedded computer systems, are in an open environment, so there will be access control problems. The Internet of Things has the advantages of accessibility and convenience, which at the same time lays hidden dangers for the security of medical data. Therefore, security and privacy are an important trend of future research. [3, 32, 33].

## 6. Conclusion

This paper conducts a bibliometric analysis of research related to machine learning and blockchain technologies' application in smart healthcare. Based on the quantitative analysis of 112 intelligent medical research literatures in the Web of Science (WOS) database, the relevant conclusions were drawn. Research hotspots in this area include machine learning in telemedicine, disease diagnosis and monitoring, blockchain technology in medical data privacy, drug supply chain management, and the role of the Internet of Things in monitoring patient's vital signs. The most researched subjects illustrate the contributions of blockchain and machine learning technologies to the world of computing, engineering, and even medicine, both now and in the future. Future research will focus on fog computing, edge computing, and machine learning methods that lead to more accurate disease prevention and treatment. As implications for practice, identifying blockchain and machine learning as key themes for the application of two emerging technologies in the field of intelligent medicine helps to understand the development of research in this field, the common themes, and background, as well as the gaps and trends in research.

The article "Literature Review on the Applications of Machine Learning and Blockchain Technology in Smart Healthcare Industry: A Bibliometric Analysis" was retracted in 2023. Reasons: unreliable results or conclusions; concerns about the data; concerns about the peer review; concerns about the citations.

Our study has two main contributions. First, in theory, we used the method of bibliometric visualization to analyze the application of ML and BC technologies in medical field. The purpose of this study was to guide the researchers in different fields to further study the ML and BC technologies in the field of smart healthcare, so that they can know which journals, authors, and articles they can refer to when studying this phenomenon. We analyzed the latest research trends based on ML and BC technology in order to provide a research direction for future research. Second, we divided the study into five clusters by clustering and revealed the substantive relationship between the clusters. Our research provided healthcare practitioners with an insight to keep ML and BC technologies fully utilized. With this study as a foundation, new research can address the lack of research and advanced knowledge in the field. We hope that future studies will provide a deeper contribution by measuring references to data obtained through Web of Science and explain the impact of the study.

## Figures and Tables

**Figure 1:** Number of documents per year from the studies.

**Figure 2:** Number of documents based on subject areas of the smart healthcare studies.

**Figure 3:** Documents based on sponsoring funding of the studies.

**Figure 4:** Number of documents by country of smart healthcare studies.

**Figure 5:** Map of hotspots.

**Figure 6:** Map of study field.

**Figure 7:** Map of research trends.

**Table 1:** The most cited papers in smart healthcare research.

	Article title	Times cited	Year	Publisher	Authors	Theme
1	ECG signal preprocessing and SVM classifier-based abnormality detection in remote healthcare applications	47	2018	IEEE Access	Venkatesan, C; Karthigaikumar, P; Paul, A; Satheeskumaran, S; Kumar, R	Machine learning & remote healthcare application

2	Bmpls: Blockchain-based multilevel privacy-preserving location sharing scheme for telecare medical information systems	32	2018	J Med Syst	Ji, YX; Zhang, JW; Ma, JF; Yang, C; Yao, X	Blockchain & Multilevel Privacy-Preserving

3	Disease diagnosis in smart healthcare: innovation, technologies, and applications	28	2017	Sustainability-Basel	Chui, KT; Alhalabi, W; Pang, SSH; de Pablos, PO; Liu, RW; Zhao, MB	Machine learning & disease diagnosis

4	A smart healthcare monitoring system for heart disease prediction based on ensemble deep learning and feature fusion	25	2020	Information Fusion	Ali, F; El-Sappagh, S; Islam, SMR; Kwak, D; Ali, A; Imran, M; Kwak, KS	Deep learning & healthcare monitoring

5	Towards a remote monitoring of patient vital signs based on IoT-Based blockchain integrity management platforms in smart hospitals	25	2020	Sensors-Basel	Jamil, F; Ahmad, S; Iqbal, N; Kim, DH	IoT-based blockchain & monitoring patient's vital sign

6	Healthchain: a blockchain-based privacy-preserving scheme for large-scale health data	25	2019	IEEE Internet of Things	Xu, J; Xue, KP; Li, SH; Tian, HY; Hong, JA; Hong, PL; Yu, NH	Blockchain & privacy health data

7	Machine learning classification of medication adherence in patients with movement disorders using nonwearable sensors	23	2015	Comput Biol Med	Tucker, CS; Behoora, I; Nembhard, HB; Lewis, M; Sterling, NW; Huang, XM	Medication adherence & machine learning

8	Recent patient health monitoring platforms incorporating internet of things-enabled smart devices	22	2018	Int Neurourol J	Kang, M; Park, E; Cho, BH; Lee, KS	Health monitoring & IoT

9	A novel medical blockchain model for drug supply chain integrity management in a smart hospital	20	2019	Electronics-Switz	Jamil, F; Hang, L; Kim, K; Kim, D	Drug supply chain integrity management & blockchain

10	A hybrid deep learning model for human activity recognition using multimodal body sensing data	20	2019	IEEE Access	Gumaei, A; Hassan, MM; Alelaiwi, A; Alsalman, H	Machine learning & body sensor

The article "Literature Review on the Applications of Machine Learning and Blockchain Technology in Smart Healthcare Industry: A Bibliometric Analysis" was retracted in 2023. Reasons: unreliable results or conclusions; concerns about the data; concerns about the peer review; concerns about the citations.

## Data Availability

The data used to support the study are available from the corresponding author upon request.
